# Acute oral toxicity of Insampaedok-san, a traditional herbal formula, in rats and its protective effects against ovalbumin-induced asthma via anti-inflammatory and antioxidant properties

**DOI:** 10.1186/1472-6882-14-365

**Published:** 2014-09-29

**Authors:** Yeji Kim, Mee-Young Lee, Ohn-Soon Kim, Woo-Young Jeon, Hyeun-Kyoo Shin

**Affiliations:** Herbal Medicine Formulation Research Group, Korea Institute of Oriental Medicine, 483 Expo-ro, Yusung-gu, Daejeon, 305-811 Republic of Korea

**Keywords:** Insampaedok-san, Safety, Cytokine, Free radical scavenging, Asthma

## Abstract

**Background:**

Insampaedok-san (ren-shen-bai-du-san in Chinese) is a traditional herbal formula widely used for the treatment of respiratory diseases in Korea and China. In this study, we investigated the acute oral toxicity of an Insampaedok-san water extract (ISSE) in rats and the antiasthmatic effects of ISSE and its mechanism in a model of asthma induced by ovalbumin (OVA) in mice.

**Methods:**

In a safety study, ISSE was administrated orally to rats of both sexes at single doses of 0 and 5000 mg/kg. We observed body weight changes, mortality, clinical signs, and gross pathological findings. In vitro antioxidant activity of ISSE was measured using 2,2-diphenyl-2-picrylhydrazyl and 2,2-azino-bis(3-ethylbenzothiazoline-6-sulfonic acid radical scavenging methods. A model of asthma was established in mice by sensitization and challenge with OVA. We assessed the levels of type 2 T-helper cytokines, chemokines, and immunoglobulin levels, using enzyme-linked immunosorbent assays, and superoxide dismutase (SOD) activity using a kit.

**Results:**

No adverse effects were observed in the acute ISSE toxicity study. ISSE showed potent free radical scavenging activity and inhibited the recruitment of inflammatory cells into the lung and mucus hypersecretion in OVA-challenged mice. ISSE significantly decreased levels of interleukin (IL)-4, IL-5, eotaxin, and OVA-specific immunoglobulin (Ig)E, and increased SOD activity.

**Conclusions:**

These results indicate that ISSE is safe for human consumption and its antiasthmatic effect is associated with the ability of ISSE to attenuate inflammation and oxidative stress.

## Background

Asthma is a chronic inflammatory disease of the airways. The pathological changes in asthma include airway obstruction, mucus hyperproduction, and increased infiltration of inflammatory cells, including eosinophils, mast cells, and lymphocytes [1]. Type 2 T-helper (Th2) cells activated by allergens play a pivotal role in the development of asthma. Activated Th2 cells produce various cytokines, including interleukin (IL)-4, IL-5, and IL-13, which induce activation and recruitment of inflammatory cells, and overproduction of mucus, during the inflammatory process in asthma. Th2 cytokines can also lead to the production of allergen-specific immunoglobulin (Ig)E antibodies by B cells [2, 3]. Inflammation in the airways induces oxidative damage. Activated immune cells, such as macrophages, neutrophils, and lymphocytes, release reactive oxygen species (ROS) [4]. Airway cells and tissues are also exposed to exogenous ROS stress from air pollutants and cigarette smoke [5]. Increased oxidative stress exacerbates inflammation by inducing proinflammatory mediators and contributes to the development of asthma [6].

Insampaedok-san (ISS; ren-shen-bai-du-san in Chinese) is a traditional herbal formula widely used for the treatment of common cold-related symptoms in Korea and China [7]. There are several case studies demonstrating the efficacy of ISS for respiratory diseases, such as the common cold and asthma [8–11]. It has been reported that the administration of this herbal medicine effectively attenuates symptoms of asthma and reduces the rate of relapse [10, 11]. Our previous *in vitro* study revealed that Insampaedok-san has anti-inflammatory, anti-allergic, and anti-obesity effects [12]. Therefore, in the present study, we performed an acute oral toxicity study of ISS in rats to establish a safety profile for ISS. In addition, we examined the antioxidant activity of ISS and its antiasthmatic effects by using a mouse model of asthma induced by ovalbumin (OVA) in vivo to investigate the mechanism underlying the effectiveness of ISS in the treatment of asthma.

## Methods

### Preparation of the Insampaedok-san water extract (ISSE)

ISSE was prepared in our laboratory from a mixture of chopped crude herbs (Table 1). Before performing the study, the identity of each crude herb was confirmed by Professor Je-Hyun Lee of Dongguk University (Gyeongju, Korea). ISSE was extracted in distilled water at 100°C for 2 h. The solution was evaporated to dryness and freeze-dried (extraction yield: 20.89%).

**Table 1:** **Composition of ISSE**

Scientific name	Part of use	Amount (g)	Company of purchase	Source
*Panax ginseng*	Radix	3.75	Omniherb	Geumsan, Korea
*Bupleurum falcatum*	Radix	3.75	HMAX	China
*Angelica decursiva*	Radix	3.75	HMAX	China
*Ostericum koreanum*	Radix	3.75	HMAX	China
*Aralia continentalis*	Radix	3.75	Omniherb	Yeongcheon, Korea
*Citrus aurantium*	Fructus	3.75	HMAX	China
*Platycodon grandiflorum*	Radix	3.75	Omniherb	Yeongcheon, Korea
*Cnidium officinale*	Rhizoma	3.75	Omniherb	Yeongcheon, Korea
*Poria cocos*	Hoelen	3.75	HMAX	China
*Glycyrrhiza uralensis*	Radix	3.75	HMAX	China
*Mentha arvensis*	Herba	3.75	Omniherb	Yeongcheon, Korea
*Zingiber officinale*	Rhizoma	3.75	Omniherb	Yeongcheon, Korea
Total amount		45.00		

### Animals for acute oral toxicity study

Twenty Sprague Dawley (SD) rats (5 weeks) of each sex were obtained from the Orient Bio Co. (Seoul, Korea). They were acclimated to laboratory conditions for 5 days and housed three per cage in an animal experiment room where the temperature was set at 23 ± 3°C, humidity at 50 ± 10%, ventilation frequency at 10–20 times per hour. They had free access to sterilized tap water and commercial rodent chow (PMI Nutrition International, USA). This study was performed at the Korea Institute of Toxicology (KIT) (Daejeon, Republic of Korea) and conducted according to guidance from the Institutional Animal Care and Use Committee at the KRICT (accredited by AAALAC International, 1998) under the GLP Regulations for Nonclinical Laboratory Studies.

In a previous experiment for dose selection, we conducted an acute toxicity study with three dose levels of 1250, 2500, and 5000 mg/kg. We found no signs of toxicity at these three dose levels. Based on these findings, we determined 5000 mg/kg as an experimental dose for the 15-day acute toxicity study. Both the ISSE group and the vehicle-only control group consisted of five rats of each sex. ISSE and distilled water (vehicle control group) were administered to rats in the treatment and control group, respectively, via oral gavage once a day and were observed for 15 days.

The general symptoms, signs of toxicity and mortality were observed over 6 h after the initiation of administration, and once a day for 15 days. The body weight of each rat was measured before the treatment and 2, 4, 8, and 15 days after treatment. At the end of the study (day 15), all rats were sacrificed by bleeding from the abdominal aorta under CO_2_ anesthesia and we performed gross observation.

### 2,2′-azino-bis(3-ethylbenzothiazoline-6-sulfonic acid) diammonium salt (ABTS) radical scavenging activity

The ABTS radical scavenging activity of the extracts was determined using a method described by Re et al. [13], with slight modifications. Briefly, ABTS radical cation was produced by reacting 7 mM ABTS solution with 2.45 mM potassium persulfate stored in the dark at room temperature for 16 h. Prior to the assay, the solution was diluted with phosphate buffered saline (PBS, pH 7.4) to an absorbance of 0.7 at 734 nm. Then, ABTS^· +^ solution was added to a 96-well plate containing samples. After 5 min of incubation, the absorbance was immediately measured at 734 nm using a microplate reader (Benchmark Plus, Bio-Rad, USA). The extent of decolorization was calculated as the percentage reduction of absorbance. The scavenging capability of test compounds was calculated using the following equation:


where A_control_ was the absorbance of the negative control, and A_sample_ was the absorbance of the standard antioxidant or extract. RC_50_ values (the concentration required for 50% reduction of ABTS radical) were calculated from the absorbance diminished by 50%.

### 2,2′-diphenyl-2-picrylhydrazyl radical (DPPH) scavenging activity

Radical scavenging activity of extracts was determined using DPPH as a free radical using the method described by Moreno et al. [14], with some modifications. Briefly, 100 μL of various concentrations of sample was added to 100 μL of DPPH solution (0.15 mM in ethanol) in a 96-well plate. After 30 min incubation in the dark at room temperature, the absorbance was measured at 517 nm. Activity of scavenging (%) was calculated using the above formula.

### Model of asthma induced by OVA and treatment

Seven-week-old female BALB/c mice, obtained from Orient Co. (Seoul, Korea), were used after 1 week of acclimation. All experimental procedures were conducted in accordance with the NIH Guidelines for the Care and Use of Laboratory Animals and were approved by Korea Institute of Oriental Medicine Institutional Animal Care and Use Committee. The animals were cared for in accordance with the dictates of the National Animal Welfare Law of Korea. Mice were divided into five groups, including a normal control group, an asthma model group, a positive control group treated with montelukast (30 mg/kg, Sigma, St. Louis, MO), and the ISSE-treated group (100 and 200 mg/kg). Briefly, mice in the asthma model group were sensitized with an intraperitoneal injection of 20 μg OVA and 2 mg aluminum hydroxide in 200 μL PBS buffer (pH 7.4) on days 0 and 14. On days 21, 22, and 23 after initial sensitization, mice were challenged with OVA (1%, w/v, in PBS) for 1 h using an ultrasonic nebulizer (NE-U12; Omron Co., Tokyo, Japan). Mice in the positive control and ISSE groups were treated orally with montelukast and ISSE (100 mg/kg and 200 mg/kg), respectively, once daily on days 18–23. Mice in the normal control and asthma model groups were given PBS. Animals were sacrificed by intraperitoneal injection of pentobarbital (50 mg/kg, Hanlim Pharm., Seoul, Korea) 48 h after the final challenge.

### Inflammatory cell counts in bronchoalveolar lavage fluid (BALF)

Mice were sacrificed with an overdose of pentobarbital 48 h after the final challenge. BALF was collected by washing lungs with ice-cold PBS (total volume of 1.8 mL) via tracheal cannulation. BALF was centrifuged and cell pellets were resuspended in 0.5 mL PBS, and cells in 100 μL of each solution spun onto a slide using a cytospin device (Hanil Science Industrial, Seoul, Korea). After the slides were dried, cells were stained using Diff-Quik Staining reagent (B4132-1A; Dade Behring, Deerfield, IL), according to the manufacturer’s instructions.

### Measurement of cytokines and chemokine levels in BALF

The concentrations of IL-4, IL-5, and eotaxin in BALF of mice were measured using enzyme-linked immunosorbent assay (ELISA) kits following the manufacturer’s instructions (BioSource International, Camarillo, CA, USA).

### Detection of OVA-specific immunoglobulin (Ig)E levels in BALF and serum

Serum was collected and stored at −70°C after centrifugation (200 *g*, 10 min). Total and OVA-specific IgE levels were measured by ELISA. Microtiter plates were coated overnight with 10 μg/mL OVA in PBS-Tween 20. After washing and blocking the plate, samples were incubated for 2 h, and then HRP-conjugated goat anti-mouse IgE was added. After washing, 200 μL of o-phenylenediamine dihydrochloride (Sigma, St. Louis, MO) was added to each well. After incubation for 10 min in the dark, absorbance was measured at 450 nm using a microplate ELISA reader.

### Measurement of superoxide dismutase (SOD) level in lung tissue

The homogenates of lung tissues were centrifuged at 12,000 *g* for 20 min to collect supernatants for determination of SOD activity. SOD activity was assayed using a kit according to the manufacturer’s instructions (Cayman, Michigan, CA). SOD activity was determined with a modified method using a NADH-phenazine methosulfate-nitroblue tetrazolium formazan inhibition reaction, which was measured spectrophotometrically at 560 nm.

### Histopathology

After BALF were obtained, lung tissue was removed, fixed with 10% (v/v) neutral buffered formalin. Tissues were embedded in paraffin, sectioned at 4 μm thickness, and stained with hematoxylin and eosin (H&E) (Sigma, St. Louis, MO) and periodic acid–Schiff (PAS) solution (IMEB, San Marcos, CA) to assess inflammation and mucus production, respectively. Tissue sections were examined microscopically.

### Statistical analysis

Data are expressed as means ± S.E.M. Statistical comparisons were made using a one-way analysis of variance (ANOVA). *P* < 0.05 was considered statistically significant.

## Results

### Acute oral toxicity study of ISSE in rats

No rats died during the 15-day acute toxicity study. There was no significant difference in body weight of either male or female rats between the ISSE-treated group and the control group during the 15-day observation period (Figure 1). No abnormal signs regarding general appearance, behavior, or nervous system were observed in rats from the ISSE-treated group compared with the control group rats. Moreover, we did not detect any clinical signs of adverse effects or any abnormal gross autopsy findings induced by ISSE treatment for 15 days.

**Figure 1:** **Changes in the body weight of rats treated with ISSE for 15 days.** Time course of mean body weight after oral administration of ISSE to male **(A)** and female **(B)** rats.

### Antioxidant activity of ISSE in vitro

To evaluate the antioxidant activity of ISSE, we tested its scavenging activities on ABTS and DPPH radicals. ABTS radical scavenging activities of ISSE are presented in Table 2 as a percentage of ABTS radical scavenging activity. ISSE showed the radical scavenging activity in a dose-dependent manner. The scavenging activities of ISSE were 18.19, 29.48, 49.98, and 71.85% at 25, 50, 100, and 200 μg/mL concentrations, respectively. The concentration required for 50% reduction (RC_50_) against ABTS radicals was 121.65 μg/mL, whereas the RC_50_ value of ascorbic acid, as the positive control, was 3.22 μg/mL. The antioxidant activities obtained for ISSE using the DPPH method are shown in Table 3. Similar to the ABTS assay, ISSE reduced the DPPH radical formation in a concentration-dependent manner. The RC_50_ for ISSE against DPPH radicals was 346.93 μg/mL, whereas the RC_50_ value of ascorbic acid was 10.43 μg/mL.

**Table 2:** **Scavenging effects of ISSE on ABTS** ^·^^+^

Herbal formula	Concentration	Scavenging effect	RC _50_^1^
	(μg/mL)	(%)	(μg/mL)
ISSE^2^	25	18.20 ± 1.33	121.65 ± 0.88
	50	29.48 ± 0.86	
	100	49.98 ± 0.61	
	200	71.85 ± 0.06	
AA^3^	1.25	21.15 ± 0.19	3.22 ± 0.06
	2.5	40.61 ± 1.44	
	5	75.86 ± 1.06	

^1^Concentration required for 50% reduction of ABTS^· +^ at 5-min reaction.

^2^Insampaedok-san and ^3^ascorbic acid.

Each value is the mean ± S.E.M. of triplicate determinations.

**Table 3:** **Scavenging effects of ISSE on DPPH**

Herbal formula	Concentration	Scavenging effect	RC _50_^1^
	(μg/mL)	(%)	(μg/mL)
ISSE^2^	50	1.55 ± 0.53	346.93 ± 3.28
	100	8.58 ± 0.59	
	200	26.48 ± 0.61	
	400	58.58 ± 0.52	
AA^3^	2.5	9.56 ± 1.26	10.43 ± 0.23
	5	24.27 ± 1.40	
	10	58.79 ± 0.70	

^1^Concentration required for 50% reduction of DPPH at 30-min reaction.

^2^Insampaedok-san and ^3^ascorbic acid.

Each value is the mean ± S.E.M. of triplicate determinations.

### Effect of ISSE on cell numbers in BALF

Inflammatory cells infiltrate the airways and secrete various cytokines and mediators that aggravate airway inflammation in asthma. The number of eosinophils and other inflammatory cells significantly increased in the BALF of OVA-challenged mice. By contrast, ISSE significantly suppressed recruitment of eosinophils and lymphocytes in the lungs (Figure 2).

**Figure 2:** **Effects of ISSE on the recruitment of inflammatory cells in bronchoalveolar lavage fluid (BALF) of mice.** Mouse BALF was collected 48 h after final OVA challenge. Cell numbers within at least five squares of a hemocytometer were counted using a light microscope. Dead cells were excluded using trypan blue staining. NC, negative control (PBS only); OVA, OVA-sensitized/challenged mice; Mon, montelukast (30 mg/kg) + OVA-sensitized/challenged mice; ISSE-100, ISEE (100 mg/kg) + OVA-sensitized/challenged mice; ISSE-200, ISEE (200 mg/kg) + OVA-sensitized/challenged mice. Significantly different from NC, ^#^ *P* < 0.05, ^##^ *P* < 0.01; significantly different from OVA, ^*^ *P* < 0.05, ^**^ *P* < 0.01.

### Effects of ISSE on inflammatory cell recruitment and mucus production in lung tissue

Inflammatory cell recruitment and mucus secretion in lung tissue were observed via microscopic examination. H&E-stained lung tissue from the OVA-challenged mice showed widespread eosinophil-rich inflammation in peribronchiolar and perivascular regions, and airspaces. Administration of ISSE attenuated inflammatory cell infiltration compared with the OVA-challenged group (Figure 3A).

In lung sections stained with PAS, mucus overproduction was observed in bronchial airways of OVA-challenged mice. The mucus staining was reduced in a dose-dependent manner in the lung tissue of mice from the ISSE-treated group (Figure 3B).

**Figure 3:** **Effects of ISSE on the recruitment of inflammatory cells to lung tissue (A) and mucus production (B).** Histological examination of lung tissues was performed 48 h after the final OVA challenge. Lung tissues were stained with H&E **(A)** and PAS **(B)**. NC, negative control (PBS only); OVA, OVA-sensitized/challenged mice; Mon, montelukast (30 mg/kg) + OVA-sensitized/challenged mice; ISSE-100, ISEE (100 mg/kg) + OVA-sensitized/challenged mice; ISSE-200, ISEE (200 mg/kg) + OVA-sensitized/challenged mice.

### Effects of ISSE on cytokines and chemokines in the BALF of OVA-challenged mice

To investigate whether ISSE affects Th2 cytokine and chemokine secretion, we measured IL-4, IL-5, and eotaxin levels in the BALF of mice. As shown in Figure 4, OVA challenge induced a significant increase in the levels of IL-4 and IL-5 in BALF. However, the levels of IL-4 and IL-5 were decreased in ISSE-treated mice. Similar to the cytokine levels, eotaxin levels increased in the BALF of OVA-challenged mice compared with those in PBS-treated mice, while the levels of eotaxin were decreased in the ISSE-treated group.

**Figure 4:** **Effects of ISSE on IL-4, IL-5, and eotaxin levels in BALF.** IL-4 **(A)**, IL-5 **(B)**, and eotaxin **(C)** levels were measured using an ELISA. NC, negative control (PBS only); OVA, OVA-sensitized/challenged mice; Mon, montelukast (30 mg/kg) + OVA-sensitized/challenged mice; ISSE-100, ISEE (100 mg/kg) + OVA-sensitized/challenged mice; ISSE-200, ISEE (200 mg/kg) + OVA-sensitized/challenged mice. Significantly different from NC, ^#^ *P* < 0.05, ^##^ *P* < 0.01; significantly different from OVA, ^*^ *P* < 0.05, ^**^ *P* < 0.01.

### Effect of ISSE on OVA-specific IgE levels in the BALF and serum

To investigate the effect of ISSE on the antibody response to allergens, the serum and BALF levels of OVA-specific IgE were measured using an ELISA. The level of OVA-specific IgE was elevated in the serum and BALF of OVA-challenged mice compared with the control group. ISSE treatment resulted in a reduction in the levels of OVA-specific IgE (Figure 5).

**Figure 5:** **Effects of ISSE on the levels of OVA-specific IgE in BALF and plasma.** OVA-specific IgE levels were measured using an ELISA. **(A)** OVA-specific IgE level in BALF **(B)** OVA-specific IgE level in serum. NC, negative control (PBS only); OVA, OVA-sensitized/challenged mice; Mon, montelukast (30 mg/kg) + OVA-sensitized/challenged mice; ISSE-100, ISEE (100 mg/kg) + OVA-sensitized/challenged mice; ISSE-200, ISEE (200 mg/kg) + OVA-sensitized/challenged mice. Significantly different from NC, ^#^ *P* < 0.05, ^##^ *P* < 0.01; significantly different from OVA, ^*^ *P* < 0.05, ^**^ *P* < 0.01.

### Effect of ISSE on SOD activity and HO-1 activity in lung tissue

To investigate the antioxidant effect of ISSE, we determined SOD activity in lung tissue. SOD activity was downregulated in mice from the asthma model group. ISSE treatment led to a marked increase in SOD activity (Figure 6).

**Figure 6:** **Effects of ISSE on SOD activity in lung tissue.** SOD activity was measured using a kit. NC, negative control (PBS only); OVA, OVA-sensitized/challenged mice; Mon, montelukast (30 mg/kg) + OVA-sensitized/challenged mice; ISSE-100, ISEE (100 mg/kg) + OVA-sensitized/challenged mice; ISSE-200, ISEE (200 mg/kg) + OVA-sensitized/challenged mice. Significantly different from NC, ^#^ *P* < 0.05, ^##^ *P* < 0.01; significantly different from OVA, ^*^ *P* < 0.05, ^**^ *P* < 0.01.

## Discussion

Traditional herbal medicine has a history of thousands of years and is still widely used in Korea and China. The evolution of traditional herbal medicine is based on observations and practical experience accumulated from millions of practitioners for thousands of years [15]. Because traditional herbal medicine does not have its own history of scientific development, there is little scientific research conducted on the safety of herbal formulas. Herbal medicines have often been provided to humans without scientifically rigorous toxicity testing. Recently, adverse effects of herbal medicines have been reported [15, 16]. Therefore, herbal medicine toxicity studies are needed to evaluate their safety. In the present study, we performed an acute oral toxicity study of ISSE, which is used often in respiratory diseases. ISSE was given orally to SD rats of both sexes at dose levels of 0 and 5000 mg/kg and they were observed for 15 days. Our results showed that no deaths occurred in either the vehicle-only control group or the ISSE group. The administration of ISSE did not cause an increase or decrease in rat body weight, when compared with the control group. In addition, there were no abnormal changes in clinical signs or gross observation. Overall, ISSE did not cause any adverse effects in this study; therefore, the LD_50_ of ISSE was considered to be over 5000 mg/kg for oral administration in rats.

ISS has been widely used for thousands of years in China and Korea to treat patients with respiratory diseases. Clinical trials show that ISS has a beneficial effect on the treatment of asthma [10, 11]. To evaluate its antiasthmatic effects, we performed an *in vitro* study on free radical scavenging activities of ISS and an in vivo study using a model of asthma induced by OVA in mice. Oxidative stress is a major feature of asthma. Many investigators have reported that increased levels of ROS in the asthmatic inflammatory process aggravate airway inflammation and damages molecules, such as proteins, DNA, and lipids [17, 18]. It has therefore been suggested that a combination of antioxidants may have positive impact on the treatment of asthma [4]. ISS is composed of 12 herbs, Radix Ginseng, Bupleuri Radix, Angelica decursiva Radix, Osterici Radix, Aralia continentalis Radix, Aurantii Fructus Immaturus, Platycodonis Radix, Cnidii Rhizoma, Poria Sclerotium, Glycyrrhizae Radix et Rhizoma, Menthae Herba, and Zingiberis Rhizoma Crudus. Also, ISS is composed various compounds such as liquiritin, ferulic acid, naringin, hesperidin, neohesperidin, and glycyrrhizin. Several components of ISS, such as Ginseng Radix [19], Aralia continentalis Radix [20], Aurantii Fructus Immaturus [21], Platycodonis Radix [22], and Cnidii Rhizoma [23], have been reported to possess antioxidant effects. Therefore, we investigated the total free radical scavenging activity of ISSE using DPPH and ABTS assays, which involve a hydrogen atom transfer reaction and electron transfer process, respectively [24]. As shown in the results, ISSE showed both DPPH and ABTS radical scavenging activities. Shanmugasundaram et al. have reported that excessive superoxide (O_2_^· −^) and hydroxyl (^·^OH) radical and reduced free radical scavengers (vitamin C, E, glutathione) and antioxidant enzymes (SOD, glutathione peroxidase, catalase were observed in the blood of asthmatic children during asthmatic episodes and interictally [25]. Our results indicate that ISSE is a potential source of natural antioxidant, which might be helpful in lowering oxidative stress.

We investigated the antiasthmatic effects of ISSE and its possible mechanism using a model of asthma induced by OVA in mice. ISSE markedly inhibited infiltration of inflammatory cells and overproduction of mucus in lung tissue. In addition, ISSE treatment resulted in a reduction in the levels of IL-4, IL-5, and eotaxin in BALF, and OVA-specific IgE, both in BALF and serum. ISSE increased SOD activity in lung tissue.

The major feature of asthma is an airway inflammation, in which CD4 T-lymphocytes, eosinophils and mast cells are predominantly involved [26]. ISSE mainly decreased the numbers of lymphocytes, which regulate other effector cells in the pathogenesis of asthma [27], and eosinophils, which reflect asthmatic activity and severity of asthma [27, 28], in BALF. This reduction of lymphocytes may be related to the inhibitory effects of ISSE on IL-4, IL-5, and eotaxin, which induce migration and recruitment of these cells to the airways. IL-4 promotes inflammation by inducing the differentiation of Th2 cells, and expression of ICAM-1 and VCAM-1 on endothelial cells, which increases lung cell infiltration [29, 30]. IL-5 induces growth, maturation, activation, migration, and survival of eosinophils [31]. IL-5 mRNA levels in asthmatics has a high correlation with eosinophils, airway hyperresponsiveness, and exhaled nitric oxide levels, which reflect airway inflammation [32]. Eotaxins are potent eosinophil chemoattractants stimulated by IL-4, IL-5, and IL-13 [33]. Therefore, the inhibition of eosinophil infiltration may result from less production of eotaxin and IL-5 after administration of ISSE.

Th2 cytokines are also involved in airway hyperresponsiveness and mucus production [34]. IL-4 stimulates IgE production from B lymphocytes [29]. Antigen-specific IgE binds to receptors on mast cells and sensitizes them to release mediators [35]. Activated mast cells produce diverse mediators and cytokines, which promote a hypersensitivity response characterized by contraction of bronchial smooth muscle, mucosal edema, and mucus hypersecretion [36]. Mucus hypersecretion, an important feature of asthma, is induced by eosinophils and mast-cell products [37] and goblet-cell metaplasia [34]. IL-4 and IL-5 lead to activation and infiltration of inflammatory cells. Moreover, IL-4 has the ability to differentiate airway epithelial cells into mucus-producing goblet cells [38]. In the present study, ISSE decreased OVA-specific IgE levels and mucus overproduction; this finding is consistent with its effect on Th2 cytokines.

Activated inflammatory cells can produce O_2_^· −^ and several inflammatory mediators that stimulate or promote ROS generation, which causes direct damage to tissue and cells [39] and aggravates inflammation by activation of nuclear factor kappa-B (NF-κB) [40]. SOD, an antioxidant enzyme, protects the airway from oxidant stress. However, SOD activity decreased in the oxidant-rich environment of asthma, which contributes to airway remodeling and hyperreactivity of asthma [41]. We show here that ISSE increased SOD activity compared with OVA group. This further supports that the antiasthmatic effects of ISSE are at least partially mediated by its antioxidant activity.

This finding indicates that ISSE enhances SOD production, which might mediate inhibitory effects of ISSE on inflammation and produce synergistic effects for the treatment of asthma through its antioxidant activity.

## Conclusions

The acute oral toxicity study in rats showed no adverse effects of ISSE up to a dose level of 5000 mg/kg in rats. The present study suggests that the beneficial effect of ISSE on asthma is associated with its antioxidant and anti-inflammatory activities. ISSE has free radical scavenging activity in vitro, and enhances SOD activity in lung tissue in a model of asthma in mice. ISSE suppresses inflammation induced by asthma by reducing infiltration of inflammatory cells, production of Th2 cytokines, chemokine, and antigen-specific IgE, and attenuating mucus hypersecretion. This study provides information regarding the safety and mechanism of antiasthmatic effects of ISSE. However, further research on constituents compounds’s activity and chronic toxicity are required.
